The article "Adaptor Protein Complex 1 Sigma 3 Is Highly Expressed in Glioma and Could Enhance Its Progression" was published in 2021. Journal: Comput Math Methods Med.

# Adaptor Protein Complex 1 Sigma 3 Is Highly Expressed in Glioma and Could Enhance Its Progression

**DOI:** 10.1155/2021/5086236

**Published:** 2021-07-29

**Authors:** Tingting Ye, Yifei Cheng, Chao Li

**Affiliations:** ^1^Department of Neurosurgery, The First Affiliated Hospital of Anhui Medical University, China; ^2^Department of Anesthesia, Huashan Hospital, Fudan University, China

## Abstract

**Introduction:**

Glioma is the widely occurring deadly neoplasm induced by glial cell canceration in the central nervous system, including the brain and spinal cord. The function of AP1S3 is special in numerous diseases, but its exact role in glioma remains unknown.

**Methods:**

Bioinformatics analysis was performed at the beginning. Based on TCGA database, differentially expressed genes were obtained. Protein-protein interaction (PPI) network analysis is performed by STRING. The annotation, visualization, and synthesis (DAVID) discovery database program was used for gene ontology enrichment analysis and Kyoto Encyclopedia of Genes and Genomes pathway analysis. The Kaplan-Meier curve was plotted to determine the prognostic value of AP1S3 Also, *in vitro* experiments were conducted in our research.

**Results:**

4370 differentially expressed genes were identified. 215 key genes were screened by protein-protein interaction (PPI) analysis; AP1S3 had a higher degree. The top five enriched pathways related to AP1S3 contain protein processing in the endoplasmic reticulum (ER), extracellular matrix receptor (ECM receptor) interaction, focal adhesion, advanced glycation end product (AGE) receptor for AGE (RAGE) signaling pathway in diabetic complications, and mRNA surveillance pathway. Additionally, the AP1S3 level was dramatically upregulated in glioblastoma (GBM) samples, but greatly reduced in low-grade glioma (LGG) samples when compared to that in normal tissues. The Kaplan-Meier curve data showed that AP1S3 was closely related to the disease-free survival (DFS) of glioma. Our data suggested that the expression of AP1S3 was increased in glioma in comparison with normal tissues, in line with the data of clinical samples. What was more, our data demonstrated that the reduction of AP1S3 in glioma cells could result in the inhibition of cell proliferation, invasion, and migration.

**Conclusion:**

Collectively, our results implied that AP1S3 was a promising biomarker of glioma diagnosis and displayed as an oncogene in glioma.

## 1. Background

Glioma is the commonly occurring glial neoplasm in the central nervous system [1]. The etiology stays elusive and is probably related to the exposure to high-dose ionizing radiation or rare genetic mutations [2]. Increased intracranial pressure, neurological and cognitive dysfunction, seizures, headache, jet-like vomiting, blurred vision, feeling loss, fatigue, foaming, twitching of limbs, and other symptoms are the main manifestations of glioma [3]. Glioma can cause a variety of neurological symptoms, deteriorate patients' life quality, and even threaten their lives [4]. The 5-year lethality ratio of glioma is approximately 15%-50%, depending on different conditions of diagnosis [5]. Surgery coupled with radiotherapy, chemotherapy, and other comprehensive treatments are the primary strategies for treating glioma [1, 6]. To explore novel biomarkers and therapeutic targets for glioma patients is yet urgent, even though the existing strategies could certainly prolong many patients' lifespan [7].

AP1S3 (adaptor protein complex 1 sigma 3) belongs to the adaptor protein (AP) family [8]. AP complex is a sort of transport heterotetramer, which can classify transmembrane proteins via the assembly of small transport vesicles in the cytosol [9]. Five AP complexes comprising AP1, AP2, AP3, AP4, and AP5 are screened, and the details of them are identified [10]. AP1 facilitates the transporting process of TGN to the endosome via targeting PI4KIIa and PI4KIIb [8]. Four subunits, two large subunits (G and B1), one medium subunit (M1), and one small subunit (S1), are included in AP1, similar to other AP complexes [11]. Different genes including two g (AP1G1 and AP1G2), two m1 (AP1M1 and AP1M2), and three S1 (AP1S1, AP1S2, and AP1S3) encode the four subunits in the corresponding isoforms of AP1 (Boehm and Bonifacino, 2001) [12]. Up to date, there are few reports on the role of AP1S3 in human cancers. Toda et al. revealed that highly expressed AP1S3, RACGAP1, ELOVL6, and LRRC59 exhibited significant association with weak status of prognosis in breast cancer patients [13]. Besides, Toda et al. reported that miR-204-5p directly targeted and AP1S3 further modulated RNA networks in cells of breast cancer [13]. In fact, more emerging reports suggest that AP1S3 is highly expressed in multiple cancers. Nevertheless, the function of AP1S3 in glioma is not well understood.

Here, our data revealed that AP1S3 was a glioma-specific gene. GO and KEGG analysis data demonstrated that there were top five enriched pathways related to AP1S3. Public datasets were analyzed to evaluate AP1S3 expression in LGG and GBM tissues. The link existing in the expression of AP1S3 and disease-free survival (DFS) of glioma patients was validated, so as to deeply uncover the veil of AP1S3. Besides, we attempted to evaluate the expression and function of AP1S3 in glioma. In the following studies, our data showed that AP1S3 expression was increased in the tissues and cells of glioma. Furthermore, AP1S3-mediated promotion of glioma cell proliferation and migration was perhaps conducive to finding new biomarkers or therapy for glioma patients.

## 2. Materials and Methods

### 2.1. Public Database

The Cancer Genome Atlas (TCGA) [14] covers the molecular features of more than 20,000 primary carcinomas and matches normal samples across 33 types of carcinomas. The Gene Expression Omnibus (GEO) [15] database is a sort of NCBI-executed gene expression database. The sequencing data of human glioma specimens provided by GSE4271 and TCGA were analyzed.

### 2.2. Establishment of Visualized PPI Network

The PPI network was constructed to predict the interaction between proteins. All candidate digital signatures were entered into the STRING website with a confidence level of 0.4, serving as the cutoff criterion for the construction of the producer price index network. A simple PPI table text created by STRING was visualized using cytosine (version 3.6.0, http://www.cytosine.org/). Demarcation point = 2, node score demarcation point = 0.2, k‐core = 2, and maximum depth = 100 were indicated as the demarcation point standard. Qualified hub genes were selected as potential key genes and biomarkers.

### 2.3. GO and KEGG Pathway Analysis

GO function enrichment analysis of AP1S3-associated genes was conducted using the molecular annotation system MAS 3.0 (http://mas.capitalbiotech.com/mas3/). DAVID Tools (https://david.ncifcrf.gov/home.jsp) were applied to carry out AP1S3-related pathway enrichment analysis of the KEGG pathway. *P* < 0.05 means significant difference.

### 2.4. Patients and Specimens

To determine the expression of AP1S3, 15 cases of glioma tissues and matched paracancerous tissues were obtained from Huashan Hospital (Shanghai, China). The permission of the Research Ethics Committee of Huashan Hospital was obtained for the use of human samples.

### 2.5. Cell Culture

Four glioma cell lines (SW1783, U373, SW1088, and U87) and human brain epithelial cell lines (HBEC-5I) were obtained from the Institute of Biochemistry and Cell Biology of the Chinese Academy of Sciences (Shanghai, China). They were kept in RPMI-1640 with 10% FBS (GIBCO) and 1% penicillin/streptomycin under a 37°C incubator with 5% CO_2_.

### 2.6. Cell Transfection

The specific siRNA against AP1S3 was designed and synthesized by Invitrogen's Shanghai factory. Simultaneously, negative control siRNA was synthesized accordingly. The cells were seeded and cultured in a growth medium until cell density reached up to 70%. Then, siRNAs were transfected into cells utilizing Lipofectamine 2000 reagent (Invitrogen) as the manual described. The cells were collected and subjected to corresponding experiments at 48 hours posttransfection. The negative control (NC) sequence is as follows: 5′-UUCUCCGAACGUGUCACGUTT-3′; the sequence of the effective knockout siRNA is as follows: si-AP1S3: 5′-CCGGGAAATTGTTCAGATT-3′.

### 2.7. CCK-8 Assay

Cell Counting Kit-8 (Tokyo Metropolitan Road, Japan) was applied to measure the ability of cell proliferation as the manufacturer's instruction. Briefly, approximately 5 × 10^3^ glioma cells were placed in a 96-well plate and treated with 10 *μ*l/CCK-8 solution per well for 4 hours of culture. Then, the absorbance was measured at 450 nm wavelength (OD450) in a microplate reader (Bio-Rad) and plotted with cell proliferation curve at each time point.

### 2.8. Quantitative Real-Time PCR (qRT-PCR)

Total RNA was harvested using TRIzol reagent (Invitrogen). Harvested RNA was transcribed into cDNA by PrimeScript RT Kit (Takara, USA). qRT-PCR was carried out utilizing SYBR Premix Ex Taq (Takara, USA). The detailed conditions of qRT-PCR were 95°C for 10 min, 94°C for 30 s, a total of 40 cycles, 60°C for 30 s, 72°C for 30 s, and then 72°C forever. GAPDH was applied to normalize the expression of genes. The relative AP1S3 expression was estimated by the 2^−*ΔΔ*Ct^ method. The sequences of the PCR primers are as follows: AP1S3 F primer: 5′-ctggaaggagctaaaacttgttt-3′, R primer: 5′-ctccacgtaacgatgcacaa-3′; GAPDH F primer: 5′-GGAGCGAGATCCCTCCAAAAT-3′, R primer: 5′-GGCTGTTGTCATACTTCTCATGG-3′.

### 2.9. Transwell Assay

The cells incubated in 200 *μ*l DMEM without serum were maintained in the upper compartment of a Transwell incubator (Corning, MA) for 48 hours. The cells migrating into the bottom compartment were fixed in formaldehyde for 10 minutes and stained with DAPI for 15 minutes. The number of migrated cells was counted under a microscope, and the relative percentage of migrating cells was shown as a histogram. In assessing invasiveness, the filter is precoated with matrix gel.

### 2.10. Statistical Analysis

All data derived from three separate experiments were indicated as mean ± SD. Comparisons between groups were analyzed by Student's *t*-test. One-way ANOVA was conducted to compare multiple groups. The disease-free survival (DFS) probability was analyzed by the Kaplan-Meier method, and the total survival probability and univariate analysis were calculated by the log-rank test. *P* < 0.05 means significant difference.

## 3. Results

### 3.1. Figure Out the DEGs and Construct the PPI Network

We analyzed the transcriptome data and screened 4370 differentially expressed genes (DEGs) in gliomas on the basis of TCGA database (Figure 1). After obtaining DEGs, a PPI network consisting of 215 nodes was established using a STRING database (Figure 2). The PPI network mainly included AP1S3, FLNA, CALU, ACTN1, MAPT, HSPA4, UBQLN4, RPN2, P4HB, MSN, AURKA, QGAP1, AURKA, and PGK1. These genes might be used for the identification of key biomarkers, and AP1S3 had a higher degree.

Based on the transcriptome data of 76 LGG samples and 77 GBM samples in TCGA database, 4370 DEGs were identified. Green indicates that the DEG is upregulated, red indicates that the DEG is downregulated, and black indicates that it is not expressed in one of the samples.

### 3.2. Functional Enrichment and Pathway Enrichment Analyses

We conducted enrichment GO and KEGG pathways analysis, and the data displayed that AP1S3-related enriched GO terms in biological process (BP) included neutrophil-mediated immunity, neutrophil activation, neutrophil degranulation, neutrophil activation involved in immune response, glycoprotein metabolic process, aminoglycan metabolic process, glycosaminoglycan metabolic process, membrane lipid metabolic process, glycoprotein biosynthetic process, and aminoglycan biosynthetic process (Figure 3(a)). AP1S3-related enriched GO terms in cell component (CC) contained endoplasmic reticulum lumen, cell-substrate junction, focal adhesion, secretory granule membrane, melanosome, pigment granule, lamellipodium, an integral component of endoplasmic reticulum membrane, vacuolar lumen, and lysosomal lumen (Figure 3(b)). AP1S3-related enriched GO terms in molecular function (MF) covered transferase activity (transferring hexosyl groups), hydrolase activity (hydrolyzing O-glycosyl compounds), hydrolase activity (acting on glycosyl bonds), protein disulfide isomerase activity, intramolecular oxidoreductase activity (transposing S-S bonds), cell adhesion molecule binding, UDP-glycosyltransferase activity, transferase activity (transferring glycosyl groups), carbohydrate binding, and protease binding (Figure 3(c)). AP1S3-related KEGG pathways enriched comprised protein processing in the endoplasmic reticulum, lysosome, apoptosis, proteoglycans in cancer, other glycan degradation, shigellosis, arrhythmogenic right ventricular cardiomyopathy, Salmonella infection, glycosaminoglycan biosynthesis-heparan sulfate/heparin, and sphingolipid metabolism (Figure 3(d)).

### 3.3. Highly Expressed AP1S3 in GBM Correlated with DFS

The AP1S3 gene expression map (49 LGG and 81 GBM) of 130 glioma patients was downloaded from GSE4271. The data revealed that AP1S3A expression in GBM tissue was dramatically higher compared to that in LGG tissue (Figure 4(a)). Likewise, TCGA database analysis data indicated that GBM samples highly expressed AP1S3 than LGG samples (Figure 4(b)). We performed further studies towards the comparison of AP1S3 expression between GBM/LGG samples and normal samples. TCGA database analysis data indicated that GBM samples highly expressed AP1S3 in comparison with normal samples (Figure 4(c)). Nevertheless, AP1S3 expression was lower in LGG samples than in normal samples (Figure 4(d)).

We performed Kaplan-Meier curve analysis to assess the correlation between AP1S3 expression and GBM disease-free survival using GBM TCGA database. The upper median of AP1S3 gene expression in all GBM samples was used as the cutoff point for dividing all cases into AP1S3 low group (*N* = 81) and AP1S3 high group (*N* = 81). The data showed that patients with highly expressed AP1S3 had a lower disease-free survival than patients with lowly expressed AP1S3 (Figure 4(e)). In addition, we conducted TCGA dataset analysis to verify whether higher expression of AP1S3 was associated with lower survival rates for glioma. TCGA dataset showed that patients with highly expressed AP1S3 had lower DFS than patients with lowly expressed AP1S3 (Figure 4(f)).

### 3.4. Upregulated AP1S3 Was Demonstrated in Glioma

qRT-PCR was carried out to detect AP1S3 expression in glioma tissues and adjacent normal tissues. The results displayed that compared with adjacent normal tissues, AP1S3 was highly expressed in 15 pairs of glioma samples (Figure 5(a)). To further determine the expression of AP1S3 in glioma, we also detected the expression of AP1S3 in glioma cells. The data showed that AP1S3 was markedly increased in glioma cells, especially in SW1783 and U373, compared with normal brain cells (Figure 5(b)). SW1783 and U373 cells were selected in the following studies. Our findings indicated that AP1S3 expression was increased in glioma.

### 3.5. Silenced AP1S3 Suppressed Glioma Cell Proliferation, Invasion, and Migration

Then, we explored the specific function of AP1S3 in glioma.  Figure 6(a) reveals that AP1S3 was silenced in SW1783 and U373 after transfection of si-AP1S3. Next, CCK-8 and Transwell assays were conducted to determine the impacts of ablated AP1S3 on cell proliferation, invasion, and migration. After the glioma cells were transfected with si-AP1S3, the cell proliferation ability was reduced (Figure 6(b)). Besides, Transwell assays showed that silencing AP1S3 suppressed cell migration and invasion ability (Figures 6(c) and 6(d)).

## 4. Discussion

Glioma, accompanied by a wide range of clinical behaviors, is the widely deadly neoplasm induced by glial cell canceration [16]. The prognosis of glioma is usually poor, and its morbidity and lethality are expected to be increased in the next few years, especially in developing countries [17]. The current treatment of glioma is surgery combined with chemotherapy and/or radiation therapy [18]. Nevertheless, a large number of tumors show a high degree of resistance to these interventions, and relapse is frequent since conventional therapies are not against the unique molecular characteristics of different subtypes of glioma [19]. Molecular genetics provides new insights for glioma classification and prediction of response to treatment, ranging from conventional treatments to new revolutionary treatment methods [20]. Due to the challenges of treating this cancer, it is urgent to determine additional targets that can be used as biomarkers for early diagnosis and treatment.

In this study, 4370 DEGs related to glioma were identified from the dataset analysis. Through enrichment analysis, we found that those DEGs were enriched in neutrophil-mediated immunity, endoplasmic reticulum lumen, transferase activity, protein processing in endoplasmic reticulum, and so on. At the same time, we screened 215 highly expressed genes from the PPI network for the identification of key biomarkers. Filamin A (FLNA), as a new downstream effector of mTORC2 to control the motility of GBM cells, functioned importantly in the movement and invasion of glioblastoma cells [21]. The researchers found that CALU could be used as a potential serum biomarker for glioblastoma through a significant analysis of the microarray. ACTN1, a gene related to the microenvironment, shows prognostic value in patients with malignant glioma [22]. The high expression of the microtubule-associated protein Tau (MAPT) gene is closely related to the improvement of the overall survival of LGG and the disease-free survival [23]. At present, there is no report to explore AP1S3 in glioma. Herein, we attempted to systematically investigate the function and mechanism of AP1S3 in glioma.

Gliomas contain the commonly deadly brain neoplasms in adults, accounting for 50% of all brain tumors [20]. Gliomas contain low-grade glioma (LGG) (grade II), high-grade gliomas (HGG) (grade III+IV), glioblastoma group (glioblastoma multiforme, GBM) (grade IV), and other-grade gliomas (OGG) (grade II+III) [18]. Among them, GBM is the widely occurring malignant brain neoplasm. The high invasiveness of GBM results in a higher mortality rate than any other brain tumors [24]. Therefore, it is very important to accurately predict the grade of glioma and take corresponding clinical treatment. Here, our data suggested that GBM samples highly expressed AP1S3 than LGG samples. More importantly, compared with the normal group, AP1S3 expression in GBM was greatly upregulated, while that in LGG was obviously downregulated. Additionally, our data suggested that highly expressed AP1S3 was largely associated with shorter DFS of BGM patients. These data indicate that AP1S3 is a biomarker for identifying GBM and predicting DFS of GBM.

AP1S3 was reported to be related to the development of many cancers, such as skin cancer and gliomas [8]. Li et al. revealed that reducing AP1S3 could lead to the inhibition of HCV production in Huh7.5.1 cells, subsequently hindering the incidence of liver cancer [9]. Another study demonstrated that highly expressed AP1S3 was involved in the pathogenesis of pancreatic ductal adenocarcinoma and a significant predictor of a poor prognosis of PDAC [25]. In our study, AP1S3 was detected to promote glioma cell proliferate by performing CCK-8 assay, and Transwell assay demonstrated AP1S3 enhanced the metastasis of glioma cell. These results suggested that AP1S3 probably functioned importantly in glioma occurrence and development via promoting cell proliferation, migration, and invasion.

This study has some limitations. First, the enriched GO terms and KEGG pathway related to AP1S3 obtained through bioinformatics analysis need to be evaluated through experiments. Second, more clinical samples need to be collected to further verify the clinical value of AP1S3 in GBM and LGG. In future studies, we will collect more clinical samples to explore the correlation between AP1S3 expression and clinical parameters (including clinical stage, age, and survival time) and the differential expression in GBM and LGG.

In conclusion, we conducted a bioinformatics analysis on the glioma database and screened 4370 differentially expressed genes. We established a visual PPI network and obtained 215 key genes, and AP1S3 had a higher degree. Our results showed that AP1S3 had rich functions and pathways in glioma. We proved that AP1S3 might be useful to diagnose GBM and was reported to be related to DFS of glioma patients. We further explored and discussed the function of AP1S3 in glioma cells. Our data displayed that AP1S3 was upregulated in SW1783 and U373 cells. The downregulation of AP1S3 suppressed glioma cell proliferation and migration, shedding light on the possibility of AP1S3 being the biomarker and therapy target of glioma. As far as we know, this is the first study to show that AP1S3 acts as a biomarker for glioma and predicts the poor prognosis of glioma.

## Figures and Tables

**Figure 1:** Heat map of the 4370 DEGs.

**Figure 2:** PPI networks of DEGs in glioma. The PPI network consists of 215 nodes according to the STRING database, and the AP1S3 gene is marked in red. The node represents the gene; the edge represents the interaction between the two proteins; the size of the node represents the score.

**Figure 3:** Function and pathway enrichment analysis for AP1S3-associated genes. (a–c) Enriched GO terms in biological process (BP), cell component (CC), and molecular function (MF). (d) Enriched KEGG pathways. The *x*-axis represents gene count; the *y*-axis represents GO term or enriched pathway. The color represents the *P* value.

**Figure 4:** Assessment of AP1S3A expression in GBM tissues and LGG tissues and exploration of the association between AP1S3A expression and shorter DFS of glioma patients. (a) Analysis of AP1S3 expression in LGG and GBM on the basis of the GSE4271 database. (b) Analysis of AP1S3 expression in LGG and GBM on the basis of TCGA database. (c) Analysis of AP1S3 expression in GBM and normal samples on the basis of TCGA database. (d) Analysis of AP1S3 expression in LGG and normal samples on the basis of TCGA database. (e) Kaplan-Meier (log-rank test) analysis of the correlation between AP1S3 expression and the DFS of BGM patients. (f) Kaplan-Meier (log-rank test) analysis of the correlation between AP1S3 expression and the DFS of glioma patients.

**Figure 5:** AP1S3 expression was upregulated in glioma. (a) Analysis of AP1S3 expression in glioma tissues and adjacent tissues. (b) Analysis of AP1S3 expression in glioma cells and normal brain cells. ^∗^*P* < 0.05; ^∗∗^*P* < 0.01.

**Figure 6:** Evaluation of the effects of reduced AP1S3 on cell proliferation, invasion, and migration in glioma. (a) Detection of AP1S3 expression in SW1783 and U373 cells after transfection with siRNAs. (b) Detection of cell proliferation in SW1783 and U373 cells after transfection with siRNAs. (c, d) Detection of cell invasion and migration in SW1783 and U373 cells after transfection with siRNAs. ^∗^*P* < 0.05.

## Data Availability

The datasets used and/or analyzed during the current study are available from the corresponding author on reasonable request.
